# Priority Based Congestion Control Dynamic Clustering Protocol in Mobile Wireless Sensor Networks

**DOI:** 10.1155/2015/596138

**Published:** 2015-10-04

**Authors:** R. Beulah Jayakumari, V. Jawahar Senthilkumar

**Affiliations:** Department of Electronics and Communication Engineering, Anna University, Chennai 600025, India

## Abstract

Wireless sensor network is widely used to monitor natural phenomena because natural disaster has globally increased which causes significant loss of life, economic setback, and social development. Saving energy in a wireless sensor network (WSN) is a critical factor to be considered. The sensor nodes are deployed to sense, compute, and communicate alerts in a WSN which are used to prevent natural hazards. Generally communication consumes more energy than sensing and computing; hence cluster based protocol is preferred. Even with clustering, multiclass traffic creates congested hotspots in the cluster, thereby causing packet loss and delay. In order to conserve energy and to avoid congestion during multiclass traffic a novel Priority Based Congestion Control Dynamic Clustering (PCCDC) protocol is developed. PCCDC is designed with mobile nodes which are organized dynamically into clusters to provide complete coverage and connectivity. PCCDC computes congestion at intra- and intercluster level using linear and binary feedback method. Each mobile node within the cluster has an appropriate queue model for scheduling prioritized packet during congestion without drop or delay. Simulation results have proven that packet drop, control overhead, and end-to-end delay are much lower in PCCDC which in turn significantly increases packet delivery ratio, network lifetime, and residual energy when compared with PASCC protocol.

## 1. Introduction

The high-tech advancement of microelectromechanical systems (MEMS) technology, processor designing, and wireless communication technology has made wireless sensor network (WSN) possible. It comprises tiny sensor nodes that are scattered in a physical space, organized into a cooperative network, and able to interact with their environment by sensing and monitoring physical and environmental parameters. WSNs are used in a wide range of applications from the civil sector to military [1–5]. The proposed protocol could widely be used in detecting natural disasters such as floods that occur in river originating from ice caped mountains and thus preventing life loss. Sensor nodes use wireless communication to collaborate to fulfill their tasks like reporting event to a centralized location called a base station (BS) for further processing to get valuable and needful information. The BS acts as a gateway between sensor node and end user and allows a user to productively sense and monitor from a distance.

The sensor nodes have to meet the requirements that come from the specific application such that they might have to be small, cheap, and energy efficient, they have to be equipped with the right sensors to compute and communicate the event to the base station. There are many technical difficulties which need to be overcome before WSN can be practically used. Thus network architecture needs to be modified to meet the specific needs of sensor nodes. Sensor nodes have the ability to withstand harsh environmental conditions and also due to their small size, the nodes are very constrained in all the resources. They have limited battery power, processing speed, storage capacity, and bandwidth. Because of the small battery size, the lifetime of a node is dependent on its capacity to conserve power. Depending upon the application, nodes may operate batteries for days, months, or even a year. Hence, to extend the lifetime of the sensor nodes, battery power needs to be effectively utilized. In WSNs, most of the energy consumed is during communication rather than by computation. Thus, energy efficient routing protocols need to be developed in order to effectively and uniformly utilize the energy among the sensor nodes.

The best routing protocol to suit for energy constrained network is cluster based routing protocols. These protocols organize the nodes into clusters. The number of clusters depends upon the application. There should be optimum number of clusters. Each cluster has one designated node called cluster head (CH) which is responsible for collecting data from its cluster members (CM) and transmits it to the BS. When compared to the conventional routing protocol, cluster based protocols reduce energy dissipation by eight times.

According to the nodes behaviour, WSNs can be classified as static or mobile. When compared with mobile nodes static nodes have several drawbacks [6, 7]. It is difficult to provide guaranteed optimal coverage using static nodes. Static failure node always hinders the communication in the network, which in turn affects connectivity and network quality. As the nodes move around the network, the number of packets to be routed to the BS varies drastically. This may cause congestion in the network, which results in packet loss. Time sensitive applications need data to be routed immediately without delay; otherwise the data will become useless. Network congestion can be avoided either by increasing link capacity or by controlling data rates [8–11].

To address these issues, in this paper, we proposed a novel Priority Based Congestion Control Dynamic Clustering Protocol (PCCDC) in WSNs. It is designed with the following objectives:

- To provide complete coverage and connectivity, mobile nodes are introduced and they are organized into clusters dynamically to minimize energy consumption.
- To reduce packet drop and to provide a high packet delivery ratio (PDR), congestion is computed at intra- and intercluster level using linear and binary feedback methods, respectively.
- An appropriate queue model is designed in each node to avoid prioritized packet drop or delay during congestion.

This paper is organized as follows.  Section 2 discusses the related work. In Section 3, we describe the detailed framework of the proposed PCCDC protocol. Simulation results are discussed in Section 4, and Section 5 concludes the paper along with the future scope.

## 2. Related Works

In this section, we provide a brief overview of the various research efforts carried out to control congestion in WSN. Several works related to congestion only dealt with flat topology [12–17] but cluster based congestion control protocols can solve many constraints in WSN.

Congestion control for multiclass Traffic (COMUT) [18] is a scalable and distributed cluster based mechanism for supporting multiple classes of traffic in WSN. In COMUT nodes are organized into clusters, with each cluster having the ability to monitor congestion within it. Based on the congestion estimate, the nodes in the clusters then adjust the sending rate to mitigate congestion. To do this, sentinel roles are assigned to sensor nodes to proactively monitor the network and collect statistics to infer the collective level of congestion. Regulation of sensor rates and coordination between cluster nodes is achieved by exchanging only small amounts of control packets between the sentinel sensors along flow paths. It also has the capability to operate successfully over multiple underlying routing infrastructures and fading channel conditions.

Congestion avoidance altering routing (CAAR) protocol [19] is a cluster based congestion avoidance protocol. It is introduced to reduce routing instability and to conserve energy in a resource constrained sensor network. It utilizes local data preservation strategies during congestion. Then it reallocates the traffic by altering route after detection of congestion which improves data transmission reliability. This altering routing protocol also provides load balancing in the network which in turn enhances life cycle of the clusters.

Rapid Congestion Control Algorithm (RCCA) [20] uses cluster topology for controlling congestion in WSN. It discusses the target application like earthquake and forest fire monitoring where transmitting emergency packets to the base station as soon as possible is much more important than conserving energy of the sensor node. Srinivasan and Murugappan [21] proposed a transport protocol for congestion avoidance in WSN based on cluster topology. The number of sensor nodes in each cluster depends on desired accuracy. The nodes are arranged in a tree topology in such a way that a node which is CH in one cluster can be CM in another cluster and sink can always be a root node. To avoid congestion for both continuous and event based sensor network, it uses hop-by-hop congestion control scheme to transmit data to the corresponding parent nodes until they reach the sink.

Energy efficient congestion control protocol [22] adjusts the data transport rate to minimize energy consumption. Congestion control is done using the sum of the node weights. Each node adds its weight with the received weight downstream and passes it to upstream. The source obtains sum of all weight information and uses it for adjusting the rate. Clustering algorithm to partition sensor nodes is done based on the sending rate and similarity of data obtained. After cluster formation nodes within the cluster communicate with its Cluster Head alternatively on a schedule to save energy.

Priority based application specific congestion control clustering protocol (PASCC) [23] integrates the mobility and heterogeneity of the nodes. PASCC detects congestion in WSN based on the type and priority of the captured data. CHs prioritize packets based on the distance; the farther nodes get priority over those of nearby nodes. It also makes sure the extra resources consumed by farther nodes are utilized effectively. During congestion, prioritized packets are routed to BS due to their timeliness requirements and nonprioritized packets are dropped. PASCCC achieves better performance in terms of the network lifetime, energy consumption, data transmission, and other QoS metrics.

## 3. The PCCDC Protocol

In this section, we discuss the detailed framework of our proposed PCCDC protocol for WSNs. PCCDC is a protocol that considers mobile nodes with homogeneous nature which are organized dynamically into clusters. It is capable of detecting and alleviating congestion at intra- and intercluster level using linear and binary feedback, respectively. It also uses an appropriate queue model in each node to avoid prioritized packet drop or delay during congestion. The assumptions made for the protocol design are presented below.

- Nodes are deployed randomly in the sensor field with a same set of energy level.
- Nodes are allowed to move around the sensing field at different speed to provide necessary coverage and connectivity.
- Each cluster should have only one CH. Therefore the number of CHs always determines the number of clusters.
- CMs are capable of adjusting their transmission power in order to reach their respective CH during a specific round.
- BS is always situated outside the sensing field which is mobile in nature and has the highest energy when compared with all the other nodes in the WSN.

### 3.1. Framework of PCCDC

Static WSN provides partial coverage of the sensing field. To provide complete coverage, the proposed PCCDC protocol uses mobile nodes which move around the sensing field to observe specific event that satisfies certain prespecified conditions. PCCDC is an application specific protocol which considers two application parameters, flooding (overflow of water) and temperature, which results in a multiclass traffic. Flooding is considered to happen when the temperature rises above the threshold value constantly in ice capped mountains. Since flooding occurs instantaneously, its traffic should be reported immediately to the base station. The packets in this case should be with less delay. This is called real-time packets. The real-time packets require preferential service when compared to the other. On the other hand sensing temperature and reporting to the base station happen periodically and are referred to as non-real-time traffic. In case of real-time traffic occurrence, traffic flows intersect with one another and region around the intersection creates a congestion hotspot [24]. This type of congestion is called forwarded congestion. It is difficult to identify the intersection points in forwarded congestion due to network dynamics. Dynamic clusters can handle forwarded congestion where the designated CH collects the traffic flow from its cluster members and aggregates and then communicates it to the BS. Appropriate queue models in each node provide a reliable delivery for real-time traffic when compared with non-real-time traffic.

### 3.2. PCCDC Mechanism

In this subsection, highlights of PCCDC protocol are given in consensus with congestion detection and control. It also provides an application overview, clustering methodology, queuing model, and energy consumption model.

#### 3.2.1. PCCDC: An Application Specific Protocol

PCCDC is designed to support and sense two different application parameters. Each node is equipped with two types of sensors, one to monitor flooding and the other to sense temperature. The following are the assumptions made:

- The node senses temperature and transmits them continuously to their respective CH and then to BS.
- The nodes start sensing flood only when the temperature reaches the threshold value; till then the flooding sensor remains idle.

Temperature packets have a low priority and result in a packet drop and some delay. On the other hand flood has high priority and should be reported without any delay and packet drop. When the sensed temperature *s*_*T*_ is less than the temperature threshold *T*_*t*_ value the nodes only sense temperature and update the CH. We set the value of *T*_*t*_ to 10°C. *T*_*t*_ is the minimum temperature required for flooding sensors to operate. When the sensed temperature *s*_*T*_ goes above the temperature threshold *T*_*t*_, then flooding sensor is turned on and allowed to capture flooding packets.

PCCDC is suitable for monitoring ice capped mountains with higher altitude. The ice melts when the temperature rises and water formed causes flooding in the rivers which originates from them.

#### 3.2.2. PCCDC: Clustering Operation

PCCDC is a dynamic cluster based protocol, which is iterative and provides different sets of clusters in each round. Every node maintains an update table. The update table holds information related to congestion of the neighboring nodes within the cluster. Each node computes its own weight and floods it to the neighbors which in turn update their update table. The fields in the update table are as follows:

 〈*node id, current queue length, residual energy, congestion level*〉

where* node id* is the address of the neighbor,* current queue length* is the instantaneous queue length of the node and incremented or decremented by 1 whenever a packet is getting enqueued or dequeued, respectively,* residual energy* is the remaining energy of the node, and* congestion level* is found by comparing* current queue length* and* residual energy* against status table as discussed in Section 3.2.3.

PCCDC calculates the weight of node *i* which is given in the (1) and (2). Consider the following:

(1) $$\begin{array}{c} W_{i}=\alpha *\Delta_{i}+\beta *E_{Ri}+\gamma *Q_{Li}, \end{array}$$

where, *α*, *β*, and *γ* are nonnegative weight coefficients. It is equal to 0.33. Consider the following:

(2) $$\begin{array}{c} \Delta_{i}=\left|\;d_{i}-N\;\right|, \end{array}$$

where  *d*_*i*_ is the degree of the node *i* by counting its neighbors, *N* is the maximum size of a cluster in terms of number of nodes, Δ_*i*_ is the degree difference for the node *i*, *E*_*Ri*_ is the residual energy for the node *i*, and *Q*_*Li*_ is the current queue length of the node *i*.

The nodes which have more weight in a particular region will act as a CH node for the current round. Each cluster is governed by a CH, which is responsible for gathering data produced by its CMs and detect congestion.

After CHs election, each CH broadcasts an advertisement packet to the neighbor nodes. The CHs contend for the medium using a CSMA (Carrier Sense Multiple Access) protocol with no further provision against the hidden-terminal problem. The non-CH nodes pick the advertisement packet with the strongest RSS in order to join themselves to a specific CH [18] using CSMA protocol. After a neighboring node decides to join to a specific CH, it unicasts a join-request message, which contains its identity and the identity of the specific CH. After cluster formation, it is the responsibility of a CH to allocate TDMA time slots to its members and broadcasts this in the broadcast schedule. This allows nodes to wake up only during TDMA time slot and gets an opportunity for transmitting data. Here TDMA based MAC (Medium Access Control) protocol is integrated with a simple routing protocol.

During data transmission phase, the sensed data from each CM can be forwarded to its CH node in the allocated TDMA slot. The numbers of slots assigned to CM are based on the current queue length and residual energy of the node at a particular time. Each CM can be assigned more than one slot in the current round. The communication between CH and its CMs is called intracluster communication. Then CH aggregates all the data packets transmitted by CMs to eliminate redundant packets. This reduces the number of packets forwarded to the BS, which in turn reduces energy dissipation and enhances the network lifetime. The communication between the CHs and the BS is called as intercluster communication.

The clustering period is defined as the start of the setup phase to the completion of the data transmission phase. Data aggregation is an energy efficient technique where packets from different neighbor are merged into a single packet, since it requires limited computational power and memory when compared with conventional transmission. Data aggregation gives exact information about the sensor field to the BS from where the end user can collect data. For every *n* packets received by CH during intraclustering, it only forwards *m* packets to the BS during interclustering, where *m* is much smaller than *n*. The *m* packets received in BS got a high degree of accuracy when compared with *n* packets. To balance the energy consumption over multiple nodes, the cluster head role is rotated periodically. The decision to become cluster head depends on the current buffer queue length and the residual energy at the node in PCCDC. When the node carries more space in its queue against the specified queue threshold and has more residual energy this node becomes CH for the particular round. It ensures that nodes consume energy more uniformly and try to avoid the black hole problem which increases the network lifetime.

#### 3.2.3. PCCDC: Congestion Detection and Control

Mobile nodes in PCCDC protocol introduce unbalanced clusters. Hence the number of nodes in each cluster varies considerably. The clusters which carries more nodes are called over crowed clusters; the level of congestion in these clusters is high. During a multiclass traffic, congested cluster can delay or drop packets randomly which makes the network useless.

In PCCDC congestion is computed in two levels, intracluster level and intercluster level. In intracluster level, hop-by-hop congestion detection and control with linear feedback is used. When a CM “*x*” wanted to forward packets to CH through intermediate CM “*y*,” then the node CM “*x*” would get the current queue length *Q*_*L*_ and the residual energy *E*_*R*_  of the node *y* in its update table. It is compared with the status table as shown in Table 1. The status value is derived using the current queue length *Q*_*L*_ and residual energy *E*_*R*_. Based on the status value node *x* would transmit packet to node *y*; otherwise node *x* would find another neighbor to CH or selectively drop packets. This is called linear feedback [25] where nodes proactively monitor neighbor nodes queue length and residual energy which is piggybacked in the data packet header. In order to reduce the control overhead involved in transmitting packets, binary feedback was not considered at the intracluster level. Queue in each node is bound with two threshold values lower queue threshold *Q*_TL_ and upper queue threshold *Q*_TH_ which are used to find the level of congestion.

In intercluster level, end-to-end congestion detection and control with binary feedback is used. The CH sends all the aggregated data to BS through multihop communication which may contain congested CH. In PCCDC protocol, when a CH “*x*” wants to communicate with BS through intermediate CH “*y*,” the node checks the current queue length and residual energy of CH “*y*” in its routing table. If the node *y*'s current queue length was within the specified threshold with optimal residual energy, then node *x* would transmit the packet to node *y*. Otherwise node *x* adds a congestion bit in the control packet and then finds another route to CH or selectively drops the packets. This is called binary feedback [20]. When a network consistently drops packet, congestion become apparent. Packet drops are mainly due to queue overflow. Since the queue size is substantially limited it is difficult to control the queue overflow in sensor network. Congestion is mostly associated with the queuing model of each node.

#### 3.2.4. PCCDC: Residual Energy Computation

The energy needed for routing packets depends on the residual energy at the link and at the node. It is the sum of energy at link and reciprocal energy available at the node [26]. This reciprocal function always assigns higher values to nodes having low residual energy. Consider as in Figure 1 that CM “*x*” wants to forward a packet to CH through an intermediate CM “*y*” or CM “*z*.” The node computes the residual energy between CM “*x*” and CM “*y*” and between CM “*x*” and CM “*z*” and then the node decides the best next hop neighbor to reach CH. Assume that the energy level at the link between CM “*x*” and CM “*y*” and between CM “*x*” and CM “*z*” is the same which is equal to 2. But residual energy at CM “*y*” is 1 and at CM “*z*” is 2. Therefore energy required between CM “*x*” and CM “*y*” is 2 + 1/1 = 3 and between CM “*x*” and CM “*z*” is 2 + 1/2 = 2.5. It is concluded that the nodes which have low residual energy are assigned with higher value and vice versa. Here, CM “*x*” decides to forward the packets to CH through the neighbor node CM “*z*” based on its residual energy during intraclustering. Similarly, CH node also calculates the residual energy of its neighboring CH to reach the BS with lesser residual energy during interclustering.

#### 3.2.5. PCCDC: Queue Model and Its Operation

The queue model in each sensor node plays a prominent role in the quick delivery of packets. Each sensor node has a queue to hold packets to be transmitted. Queue overflow occurs when a node receives packets with a higher data rate than it can transmit. To overcome this situation, a congestion control algorithm (Algorithm 1) can either reduce the data rate or selectively drop the packets which have lesser importance or reroute the packets through alternate path, which improves the throughput at the BS.

Figures 2 and 3 show a queue model introduced for sensor nodes in PCCDC. Each queue is bounded by two thresholds called lower threshold *Q*_TL_ and upper threshold *Q*_TH_. This facilitates the queue in three different states such as accept state, filter state, and reject state. When the queue size is less than *Q*_TL_ the queue is in accept state, where all the packets are queued. This is a congestion free state, where the queue is scheduled using a FCFS algorithm. Congestion level can be measured through an exponentially weighted moving average of the instantaneous queue length. If it exceeds lower threshold *Q*_TL_ then the behaviour of the queue changes suddenly. It wou ld selectively enqueue packets based on priority. This is the filter state which indicates congestion is going to happen in the network. Afterwards, the average queue length is updated whenever a packet is inserted into the queue. This facilitates maximizing the number of priority packets getting enqueued during congestion. During this state the queue is scheduled using a priority algorithm. However, if the queue size exceeds *Q*_TH_, then the node is said to be congested. Under this condition all packets are rejected until the current queue length *Q*_*L*_ is less than *Q*_TH_. This state is called reject state.

As a result of these packet drops, source nodes and forwarding nodes waste and exhaust their battery power and finally create a routing hole. This can reduce network lifetime and overall network connectivity. Node senses events and assigns them priorities based on the packet type not on the locations of the nodes because event occurrences are not restricted to a specific location. Priority assignment can be done by reserving one bit in each packet header.

Since PCCDC is designed with homogeneous nodes, the queue models in both CM and CH are the same but have different queuing operations. If the CM's current queue length is within the lower threshold *Q*_TL_ then all the packets are queued in FCFS. Once it exceeds lower queue threshold *Q*_TL_, then enqueue packets will contain priority bit set. In PCCDC, priority bit is set for all the real-time packets and a very low percentage of non-real-time packets. This avoids starvation problem for non-real-time packets.

High priority could be assigned to packets based on distance and sense value. In each cluster, CM far away from CH consumes more energy than nearby CM and also will expire earlier. Therefore, distance and sense value play an important role while assigning priority to packets. In WSNs, the nodes which are far away from CH could have meaningful data rather than the ones close to CH. Selective dropping or selective queuing is based on the packets proximity. The average queue length is updated after *Q*_TL_. This facilitates maximizing the number of high priority packets getting enqueued during congestion. During this state the queue is scheduled using a priority algorithm. The scheduler first schedules high priority packets *P*_*H*_ followed by *P*_*L*_ low priority packets. However, if the queue size exceeds *Q*_TH_, then the node is said to be congested. Under this condition all packets are rejected until the current queue length *Q*_*L*_ is less than *Q*_TH_.

If the current queue length of CH is within lower queue threshold *Q*_TL_ low priority packets *P*_*L*_ are queued in at the tail and high priority packets *P*_*H*_ in the head. Queue acts as a priority queue right from the beginning. When the CH's current queue length exceeds lower queue threshold *Q*_TL_ all the low priority packets *P*_*L*_ are dropped randomly based on distance and sense value. But if it exceeds *Q*_TH_ then all the packets are rejected and the control signal is sent to its parent node to reduce its sending rate. The efficiency of the PCCDC system decreases the packet drop for high priority packets *P*_*H*_ to a large extent.

## 4. Performance Evaluation

Network simulator version-2 (NS2) [27] is used to simulate the proposed PCCDC protocol. NS2 is a network simulator that is widely used in wireless environments. The simulation parameters used are summarized in Table 2. The topology used in our simulation is a random topology with random mobility model where nodes are placed at a random position within the simulation area.

### 4.1. Performance Metrics

The performance of PCCDC protocol is evaluated using the following metrics:

- *Packet drop*: it is the average number of packets dropped in the sensor network due to congestion.
- *Packet Delivery Ratio (PDR)*: it is the percentage of the total packets received successfully by the BS divided by the total packets produced by the sources.
- *Control overhead*: it is the ratio of total number of control packets used in the network to the total number of data packets received.
- *End-to-end delay*: it is the average time difference between the packets sent by the source node to the packet received by the base station.
- *Network lifetime*: it is the time taken for the energy of the first sensor node to fall from 0.5 J to zero. It is expressed in seconds.
- *Residual energy*: it is the average energy consumed by sensor node during each round throughout the network.

### 4.2. Simulation Results and Discussion

In Figure 4(a), it can be observed that PCCDC outperforms PASCC when packet drop is considered. Even though PCCDC and PASCC adopt cluster based network topology PCCDC performs better than PASCC. Since PCCDC handles intra- and interlevel congestion separately and also each node is designed with an appropriate queue model, packet drop is reduced considerably. The packet loss in PCCDC is 42.02 percent lower than PASCC. Packet drop and packet delivery ratio are inversely proportional.  Figure 4(b) demonstrates the average packet delivery ratio of random mobility model. The reduced packet loss in PCCDC results in higher packet delivery ratio of 13.62 percent over PASCC protocol.

Generally the network scales up due to dynamic environment, the number of congested nodes also increases, and in addition control packets exchanged to contain congestion considerably increase. But in PCCDC routing protocol, intercluster communication requires control packets for routing whereas intracluster communication uses linear feedback nodes that proactively listen to packets. As a result the control overhead PCCDC is 17.91 percent lower than PASCC as shown in Figure 4(c).

In cluster based protocols end-to-end delay depends on relative location between CMs and BS and the resource allocation of CHs as well. Increase in end-to-end delay is quite inevitable when the number of congested nodes increases in the network, since PCCDC protocol uses the differentiated queue model for CM and CH to reduce the end-to-end delay for real-time packets.  Figure 4(d) compares the end-to-end delay between PCCDC and PASCC. It can be understood that end-to-end delay in PCCDC is 5.07 percent less than PASCC.

Control overhead has significant effect on residual energy. In short, reduced control overhead stands for reduced residual energy which is shown in Figure 4(e). Residual energy in a node is highly determined by the energy consumed in sensing events, receiving and sending sensed data packets, and transmission of control packets. In PCCDC, the flooding sensors remain in the sleep mode until the temperature sensor exceeds threshold. Once the temperature sensor exceeds threshold, then the transmitter of flooding sensor is turned on. Until the real-time event gets detected, sensor nodes remain in the sleep mode. When the node's queue length exceeds the upper threshold, then temperature sensor also enters into sleep mode. PCCDC utilizes the limited energy of the nodes efficiently compared with PASCC. This results in 18.03% lesser residual energy in PCCDC with respect to PASCC.

The simulation was performed with 0.5 J of initial energy to calculate the network lifetime. Life time of a network is closely associated with energy consumption contributed by the protocols. If more energy is consumed the sensor nodes drain out and the network may scale down. The condition further deteriorates when congestion results in packet drop and retransmission of packets. PASCC does not choose optimal path of CHs based on the congestion estimate and hence congested CHs can easily drain out. This in turn imparts negative impact on network life time with PASCC when compared to PCCDC.  Figure 4(f) shows that PCCDC results enhanced life time of 5.62% when compared to PASCC.

### 4.3. Theoretical Analysis 

#### 4.3.1. Energy Consumption

Energy consumption can be defined as the average energy consumed by each node during the given simulation time and is expressed in Joules (J). The energy model of a PCCDC protocol for WSN is different from energy consumption model proposed in the literature [28]. In PCCDC protocol the energy consumption for sensing, receiving, and updating for a packet size *k* in bits is the same for both CM and CH node but it is different during transmission. Hence the total energy consumption of a CH node differs from that of a CM node which is derived below.

First consider the energy required for sensing a single bit in CM and CH node. It is given by

(3) $$\begin{array}{c} E_{\text{sensing}}=e_{i}*p, \end{array}$$

where *e*_*i*_ = energy consumption of a node when sensing single bit and *p* = payload of the sensed data.

The energy required for communicating is primarily due to the transceiver of the node. The two main components of a transceiver are radio electronics and power amplifier.

Generally the energy consumption in radio electronics for the packet size *k* in bits is given by

(4) $$\begin{array}{c} E_{\text{radio\_electronics}}=kE_{\text{radio}}. \end{array}$$

Also the energy consumption in power amplifier depends on the distance between transmitter and receiver. If the distance between the transmitter and receiver is less than the crossover distance *d*_cross_ then the propagation is inversely proportional to *d* ^2^ where the *f*_riss_ free space model is used; otherwise propagation is inversely proportional to *d* ^4^ where two-ray ground propagation model is used. The crossover distance is obtained using

(5) $$\begin{array}{c} d_{\text{cross}}=\sqrt{\frac{E_{\text{free\_space}}}{E_{\text{two\_ray}}}}. \end{array}$$

The energy consumption in power amplifier for the packet size *k* in bits is given by

(6) $$\begin{array}{c} E_{\text{power\_amplifier}}=\left\{\begin{array}{cc} kE_{\text{free\_space}}d^{2}, & d<d_{\text{cross}}\\ kE_{\text{two\_ray}}d^{4}, & d\geq d_{\text{cross}}. \end{array}\right. \end{array}$$

The distance *d* from CM to CH can be calculated by received signal strength indicator (RSSI). It is given in

(7) $$\begin{array}{c} d=10^{\left|RSSI-A\right|/dx}, \end{array}$$

where *A* is the received signal strength at the position which is 1 m away from the sending point. RSSI is the received signal strength indication, and *x* is the factor of path fading, which is generally 2 to 5.

Hence the energy required for transmitting the packet size *k* in bits for CM node is calculated by

(8) ETXk,d=Eradio_electronics+Epower_amplifierETXk,d=kETX_radio+kEfree_spaced2,d<dcrosskETX_radio+kEtwo_rayd4,d≥dcross.

Due to the additional data aggregation operation and long distance transmission, the energy consumption of CH is more than its CM. Therefore the energy required for both transmission and data aggregation for the packet size *k* in bits only in CH is obtained using

(9) ETXk,d=nkETX_radio+kEfree_spaced2+nkEagg,d<dcrossnkETX_radio+kEtwo_rayd4+nkEagg,d≥dcross,

where *n* is the number of CMs associated with each cluster which is given in

(10) $$\begin{array}{c} n=\frac{N}{k_{\text{optimal}}}, \end{array}$$

where  *N* is the total number of nodes in a WSN. *k*_optimal_ is the optimal number of clusters in each round. *E*_agg_ is energy consumption during data aggregation operation of CH.

But the energy required for receiving the packet size *k* in bits for both CM and CH node is the same which can be calculated using

(11) $$\begin{array}{c} E_{RX}\left(\;k,d\;\right)=E_{RX\_\text{radio}}*k. \end{array}$$

Similarly the energy required for update packet size *k* in bits for both CM and CH node is calculated using

(12) $$\begin{array}{c} E_{u}\left(\;k,d\;\right)=E_{U\_\text{radio}}*k. \end{array}$$

Therefore the total energy spent of a node *N*_*i*_ is the summation of energy consumptions during sensing, transmitting, receiving, and updating the packet size *k* in bits could be calculated by

(13) $$\begin{array}{c} E_{s}\left(\;N_{i}\;\right)=E_{TX}\left(\;k,d\;\right)+E_{RX}\left(\;k,d\;\right)+E_{u}\left(\;k,d\;\right). \end{array}$$

The energy needed for routing packets depends on the residual energy at the node *N*_*i*_ is *E*_*r*_(*N*_*i*_). Initially the energy present in the node is assumed to be 1. Energy spent for routing a packet is *E*_*s*_(*N*_*i*_). Therefore the residual energy at node *E*_*r*_(*N*_*i*_) is computed in

(14) $$\begin{array}{c} E_{r}\left(\;N_{i}\;\right)=1-E_{s}\left(\;N_{i}\;\right). \end{array}$$

## 5. Conclusion

The proposed PCCDC protocol provides complete coverage and connectivity using mobile nodes. To reduce energy consumption, nodes are organized into clusters. PCCDC clusters have two phases, namely, setup and data transmission phase. PCCDC assigns priority to real-time packets; the number of real-time packets getting dropped during congestion is reduced considerably because PCCDC handles congestion at both intra- and intercluster level separately. An appropriate queue model in CM and CH also avoids packet drop due to congestion.

In PCCDC real-time packets are captured after non-real-time packets exceed the threshold limit. This reduces the number of real-time packets being generated. Since real-time packets are time stamped, they are transmitted immediately to BS to provide higher packet delivery ratio. PCCDC also maintains coverage fidelity to ensure that packets coming from far off nodes and with more sense value are delivered immediately to avoid getting dropped. The number of control packets needed in PCCDC is much lower due to binary feedback at intercluster level thereby reducing the energy consumption which in turn increases the network lifetime. The proposed PCCDC is compared with PASCC protocols.

The proposed protocol reduces the energy consumption but at the same time incurs a slight time delay due to dynamic clustering during emergency situations. To address this time delay, it is proposed to handle the data transmission phase of PCCDC in two different situations. During normal situation CHs alone participate in data transmission to BS and under critical situation data can be transmitted through a minimum number of nodes which are surrounding the event.

## Figures and Tables

**Figure 1:** Residual energy computation.

**Figure 2:** Queuing model of a CM sensor node.

**Figure 3:** Queuing model of a CH sensor node.

**Figure 4:** Performance comparison of PCCDC and PASCC protocol against simulation time.

**Algorithm 1:** Algorithm for processing packets in CM and CH node.

**Table 1:** Status table.

Status	Description
0	*Q*_*L*_ < *Q*_TL_ with high *E*_*R*_ ready to forward
1	*Q*_*L*_ < *Q*_TL_ with medium *E*_*R*_ ready to forward
2	*Q*_*L*_ < *Q*_TL_ with low *E*_*R*_ forward packets based on priority
3	*Q*_*L*_ > *Q*_TL_ && *Q*_*L*_ < *Q*_TH_ with high *E*_*R*_ forward packets based on priority
4	*Q*_*L*_ > *Q*_TL_ && *Q*_*L*_ < *Q*_TH_ with medium *E*_*R*_ forward packets based on priority
5	*Q*_*L*_ > *Q*_TL_ && *Q*_*L*_ < *Q*_TH_ with low *E*_*R*_ forward packets based on priority
6	*Q*_*L*_ > *Q*_TH_ with high *E*_*R*_ drop packets
7	*Q*_*L*_ > *Q*_TH_ with medium *E*_*R*_ drop packets
8	*Q*_*L*_ > *Q*_TH_ with low *E*_*R*_ drop packets

**Table 2:** NS-2 simulation parameters.

Parameter	Value
Area of sensor field	1200 m × 1200 m
Number of sensor nodes	150
Radio range of a sensor node	200 m
Propagation model	Two-Ray ground
Transmit power	0.660 W
Receive power	0.395 W
Transmission range	45 m
Node placement	Random
Traffic type	CBR (UDP)
Packet size	64 bytes
Number of BS	1
MAC protocol	MAC/802.11
